The article "CRISPR/Cas9-Mediated OC-2 Editing Inhibits the Tumor Growth and Angiogenesis of Ovarian Cancer" was retracted in 2021. Reason: manipulated images.

# CRISPR/Cas9-Mediated OC-2 Editing Inhibits the Tumor Growth and Angiogenesis of Ovarian Cancer

**DOI:** 10.3389/fonc.2020.01529

**Published:** 2020-09-02

**Authors:** Tongyi Lu, Ligang Zhang, Wenhui Zhu, Yinmei Zhang, Simin Zhang, Binhua Wu, Ning Deng

**Affiliations:** Guangdong Province Engineering Research Center for Antibody Drug and Immunoassay, Department of Biology, Jinan University, Guangzhou, China

**Keywords:** ovarian cancer, OC-2, CRISPR/Cas9, apoptosis, tumor angiogenesis

## Abstract

Ovarian cancer is the leading cancer-related cause of death in women worldwide. It is of great relevance to understand the mechanism responsible for tumor progression and identify unique oncogenesis markers for a higher chance of preventing this malignant disease. The high-expression OC-2 gene has been shown to be a potential candidate for regulating oncogenesis and angiogenesis in ovarian cancer. Hence, we wished to investigate the impact of OC-2 gene on ovarian cancer aggressiveness. CRISPR/Cas9, a gene editing tool, allows for direct ablation of OC-2 at the genomic level, and we successfully generated OC-2 KO cell lines from SKOV3 and CAOV3 cells. In an apoptosis assay, OC-2 KO induced the apoptosis activation of tumor cells, with the up-regulation of Bax/Caspase-8 and the down-regulation of Bcl-2. Consequently, the proliferation, migration, and invasion of OC-2 KO cell lines were significantly inhibited. Assays of qRT-PCR and Western blotting showed that the expression levels of pro-angiogenic growth factors VEGFA, FGF2, HGF, and HIF-1α and the activation of Akt/ERK pathways were significantly down-regulated at the loss of OC-2. In the xenograft model, OC-2 KO potently suppressed the subcutaneous tumor growth, with the inhibition exceeding 56%. The down-regulation of CD31 and relevant pro-angiogenic growth factors were observed in OC-2 KO tumor tissues. Taken together, OC-2 depletion negatively regulated the ovarian cancer progression possibly by apoptosis activation and angiogenesis inhibition. This work revealed a pivotal regulator of apoptosis and angiogenesis networks in ovarian cancer, and we applied the CRISPR/Cas9 system to the transcription factor pathway for developing a broad-acting anti-tumor gene therapy.

## Introduction

Ovarian cancer is one of the most common types of malignancy for females, after cervical and endometrial cancer (1, 2). Since there are little typical symptoms at the early stage of ovarian cancer, patients at the late stage will be extremely hard to treat due to extensive abdominal metastasis (3). The key biomarkers for ovarian cancer diagnosis and treatment are demanded in spite of different heterogeneity and genotypes (4, 5). Meanwhile, the development of ovarian cancer would be inconceivable without microvessels providing nutrients and transferring metabolins (6). In the tumor environment, tumor and endothelial cells secrete various vascular factors to aggravate tumor angiogenesis, including vascular endothelial growth factor A (VEGFA), fibroblast growth factor-2 (FGF2), platelet-derived growth factor subunit A (PDGFA), hepatocyte growth factor (HGF), and hypoxia-inducible factor-1α (HIF-1α) (7–9). Currently, it has been the focus to down-regulate angiogenesis in cancer treatment through targeting pro-angiogenic growth factors (10). However, the anti-angiogenic strategies based on the blockade of single pathway resulted in modest and transient benefit in some clinic trials (11, 12). Therefore, we are committed to figuring out the upstream targets that can control the angiogenesis networks in ovarian cancer.

The article "CRISPR/Cas9-Mediated OC-2 Editing Inhibits the Tumor Growth and Angiogenesis of Ovarian Cancer" was retracted in 2021. Reason: manipulated images.

In our previous research, ONECUT Homeobox 2 gene (OC-2) was highly expressed in ovarian cancer tissues and cell lines than the normal, suggesting that OC-2 might play a pivotal role in ovarian cancer progression (13). OC-2 is a novel gene discovered in 1999 and belongs to ONECUT transcription factor family (14). The protein level of OC-2 is tissue-specific, with the strongest expression detected in human liver and skin. Margagliotti found that OC-2 was involved in the differentiation of liver organ and the regulation of TGF-β signaling pathway for hepatocyte metastasis, thereby controlling the initial liver development (15). Also, high expression of OC-2 was observed in the brain, hepatocellular, lung, colon, bladder, and prostate carcinoma, suggesting its important role in tumor progression. OC-2 had been proven to be a transcription factor that played a key role in tumor cell proliferation, metastasis, and oncogenesis (16–18). Zhang introduced the idea that OC-2 was up-regulated in hepatocellular carcinoma and partially acted as a tumor promoter through the Akt/ERK pathways (19). It was demonstrated that the epigenetic of bladder cancer could be analyzed by the OC-2 expression status, with high sensitivity and specificity (16). However, our knowledge about the function of OC-2 in ovarian cancer is still very limited, especially regarding to mechanism of OC-2 regulating the tumor growth and angiogenesis networks. Therefore, we expected to knock out the OC-2 gene using CRISPR/Cas9 system to totally investigate its functions in ovarian cancer.

Types of cell death are classified into apoptosis, necrosis, autophagy, pyroptosis, and so on (20, 21). Among them, apoptosis plays an important role in tissue differentiation, organ development, and general homeostasis. As new cells occur, aging, and mutated cells will be cleared by apoptosis in extrinsic and intrinsic manners (22). The extrinsic apoptosis is triggered by death receptor, which activates intracellular signal cascades and sequential caspases (23). In contrast, the intrinsic apoptosis in response to cellular stresses can activate caspases via the apoptosis factors released by mitochondria (24). The mitochondrial pathway is mainly regulated by the relative levels of the Bcl-2 superfamily, including anti-apoptotic and pro-apoptotic protein members (25). The members of Bcl-2 superfamily are divided into anti-apoptotic Bcl-2, pro-apoptotic Bax/Bak, and pro-apoptotic BH3-only family, which initiate and limit the mitochondria-dependent caspase activation in a balance (26–28). Dysfunction of apoptosis can make cell growth out of control, resulting in vicious transformation to tumor cells. In this process, overactive oncogenes like growth factors not only promote tumor growth but also suppress apoptosis of tumor cells as negative regulators (29). As for apoptosis, strategy of tumor therapeutics can focus on reconstructing the apoptotic signaling system, including down-regulating the expression of survival genes and activating the expression of death genes in tumor cells.

The article "CRISPR/Cas9-Mediated OC-2 Editing Inhibits the Tumor Growth and Angiogenesis of Ovarian Cancer" was retracted in 2021. Reason: manipulated images.

In this study, we needed to generate the stable CRISPR/Cas9-driven OC-2 KO cell lines of SKOV3 and CAOV3 cells. We focused on the role of OC-2 in tumor cell apoptosis, especially the expression status of pro-apoptotic genes and anti-apoptotic genes. Assays of CCK-8, wound healing, migration, invasion, and xenograft model were conducted to investigate the functions of OC-2 in tumor growth. *In vitro* and *vivo* experiments were performed to investigate the tumor angiogenesis and the expression status of pro-angiogenic growth factors at the loss of OC-2. Our results would offer a new understanding of OC-2 in regulating tumor growth and angiogenesis, which might help reveal the mechanism of OC-2 in ovarian cancer for reference in the future.

## Materials and Methods

### Cell Culture

The human ovarian cancer cell lines SKOV3 cells, CAOV3 cells, and human embryonic kidney cells (HEK293T) were obtained from the Shanghai Institute of Biochemistry and Cell Biology, Chinese Academy of Sciences. All the cells were cultured in high glucose Dulbecco's modified Eagle's medium (DMEM, Invitrogen, New York, NY, USA) supplemented with 10% fetal bovine serum (FBS, Hyclone, Logan, UT, USA) and 100 U/ml penicillin/streptomycin (Gibco, Langley, OK, USA). All the cells were incubated in a 5% CO_2_ incubator at 37°C.

### Plasmid Constructs

Based on the CDS analysis of human OC-2 gene, exon 1 (Table S1) was selected as the knockout position. Three targeted sgRNAs were obtained using a common CRISPR design tool (http://crispr.mit.edu/). The sgRNAs were synthesized by Sangon Biotech (Shanghai, China) and inserted into LentiCRISPRv2 vector at *Bsm*BI sites (Table S2), followed by enzyme validation.

The article "CRISPR/Cas9-Mediated OC-2 Editing Inhibits the Tumor Growth and Angiogenesis of Ovarian Cancer" was retracted in 2021. Reason: manipulated images.

### Lentivirus Infection

Using a 100-mm dish, 293T cells (5 × 10^4^ cells/ml) were cultured in 7 ml of DMEM supplemented with 10% FBS and 100 U/ml penicillin/streptomycin. Before infection, the medium was replaced by basal DMEM. Lentivirus together with recombinant plasmid LentiCRISPRv2 (4 μg) and packaging vectors psPAX2 (3 μg) and pMD2G (1 μg) were mixed with 24 μl of FuGENE6 Transfection Reagent (#E2691, Promega, Madison, WI, USA) and basal DMEM (total 200 μl) and incubated at 37°C for 30 min. 293T cells were incubated with the lentivirus for 6 h, and the medium was replaced by DMEM supplemented with 10% FBS and 100 U/ml penicillin/streptomycin. The lentivirus solution was collected and concentrated by an ultra-concentrator (100 KD) at 4,000 *g*, 4°C for 30 min. SKOV3 and CAOV3 cells (3 × 10^5^ cells/well) were cultured in six-well plates for another 24 h and the cells were incubated with puromycin at the concentration from 0 to 4 μg/ml for 4 days to figure out the minimum lethal dose. Then, polybrene and the lentivirus were added to infect SKOV3 and CAOV3 cells and the medium was replaced by DMEM supplemented with 10% FBS and 100 U/ml penicillin/streptomycin 24 h later.

### Clonal Isolation of CRISPR-Edited Cells

The infected cells were cultured in the medium containing puromycin (1.5 μg/ml) to achieve stable cells expressing Cas9. The survival cells were subjected to limiting dilution until single colonies were isolated. The OC-2 KO cells were verified by Western blotting, sequencing, and Cruiser^TM^ cleavage assays.

### qRT-PCR

Total RNA was extracted from the OC-2 KO cell lines and the reverse transcription was subjected to ReverTra Ace qPCR RT Kit (#FSQ-101, TOYOBO, Osaka, Japan). Subsequently, the qRT-PCR procedures were conducted with RT-PCR Reaction Mix (#TSE201, QINGKE, Beijing, China) through BIO-RAD CFX96 Cycler. Data were analyzed according to the 2^−ΔΔCT^ method and the primer sequences for mRNA detection are listed in Table S3.

### Western Blotting

Total protein was extracted from OC-2 KO cell lines with cell lysis buffer containing protein inhibitor, PMSF, and phosphatase inhibitor (#P0013, Beyotime Biotechnology, Jiangsu, China). Each sample of 30 μg of protein was separated on SDS-PAGE gel and transferred to PVDF membrane (#IPVH00010, Millipore, Bedford, MA, USA), followed by 1-h 5% nonfat milk blocking treatment (37°C). The primary antibodies rabbit monoclonal anti-t/p-Akt (#4691, 1:1000, #4060, 1:2000), anti-t/p-ERK1/2 (#4695, 1:1000, #4370, 1:2000), and anti-GAPDH (#5174, 1:1000) were purchased from Cell Signaling Technology (Danvers, MA, USA), and rabbit polyclonal anti-OC-2 (#ab28466, 1:1500) was purchased from Abcam (Cambridge, USA). The secondary antibody HRP-conjugated goat anti-rabbit IgG (#7074, 1:1000) was obtained from Cell Signaling Technology. After several washings, the blots were detected using super ECL plus (#WBKLS0100, Millipore) and the signal intensities were analyzed by ImageJ software.

The article "CRISPR/Cas9-Mediated OC-2 Editing Inhibits the Tumor Growth and Angiogenesis of Ovarian Cancer" was retracted in 2021. Reason: manipulated images.

### Apoptosis Assay

Cells (1 × 10^6^/well) were cultured for a further 24 h and then fixed with 70% ethanol overnight at 4°C. The fixed cells were stained with Annexin V-fluorescein isothiocyanate (FITC) and propidium iodide (PI, #KGA107, Keygen Biotech, Jiangsu, China) at 37°C for 30 min. After several washings, the cells were detected by FACS (BD Bioscience, San Jose, CA, USA) and the results were analyzed by FlowJo software.

### CCK-8 Assay

The OC-2 KO cell lines (2.5 × 10^3^ cells/well) were transferred into 96-well plates, and CCK-8 solution (#CK04, Dojindo, Kumamoto, Japan) of 10 μl was added 24, 48, and 72 h later. The absorbance at 450 nm was read by a microplate reader (BioTek Instruments, Winooski, VT, USA).

### Wound-Healing Assay

The OC-2 KO cell lines (3 × 10^5^ cells/well) were added into six-well plates, and the monolayer cells were scraped in a straight line using a pipette tip. The scratches were washed to remove the detached cells and incubated with DMEM supplemented with 0.5% FBS. The photographs were taken 24 h later under an inverted microscope (Olympus, Tokyo, Japan). The blank areas in the defined site were measured by ImageJ software. The recovery rates were counted by dividing the widths of the initial and final wounds.

### Migration and Invasion Assays

The migration and invasion abilities of the OC-2 KO cell lines were evaluated by the Transwell system (#353097, BD Bioscience) in 24-well plates. Matrigel (#356234, BD Bioscience) was only used in the invasion assay. The cells (2 × 10^4^cells/well) suspended in 200 μl of basal DMEM were transferred into the upper chamber while 650 μl of DMEM supplemented with 10% FBS was added in the bottom. After 24 h, the residual cells on the inner surface were removed and the migrated cells were fixed with 70% ethanol and stained with 0.1% crystal violet. The photographs were taken under an inverted microscope and the migration and invasion abilities were analyzed in five random fields by ImageJ software.

### Mice and Xenograft Model

The BALB/c nude mice (female, 6 weeks) were purchased from Beijing Huafukang Biological Co., Ltd. The mice were subcutaneously inoculated with OC-2 KO cell lines (1 × 10^6^ cells/mouse) in the right shoulders. SKOV3 and CAOV3 cells served as the control. Tumor growth was measured by a caliper every 3 days and tumor volume was calculated by means of caliper measurements (Formula: π × Length × Width^2^/6). The expression of CD31, OC-2, VEGFA, and HIF-1α in the tumor tissues was subjected to IHC assay. To assess the effect of OC-2 knockout on tumor growth, the tumor volumes at different times were analyzed by mixed-effects models for repeated-measures ANOVA.

The article "CRISPR/Cas9-Mediated OC-2 Editing Inhibits the Tumor Growth and Angiogenesis of Ovarian Cancer" was retracted in 2021. Reason: manipulated images.

### Immunohistochemistry (IHC)

Tumor tissues stripped from the xenograft model were fixed in 4% paraformaldehyde and embedded in paraffin. To repress the endogenous peroxidase activity, the tumor sections were treated with 10 mM sodium citrate buffer (pH 6.0) and 3% H_2_O_2_ after deparaffinization. Then, 5% BSA and 0.05% Triton X-100 were added for blocking treatment. The primary antibodies rabbit polyclonal anti-OC-2 (1:500) and anti-CD31 (#ab28364, 1:50) and rabbit monoclonal anti-VEGFA (#ab52917, 1:100) and anti-HIF-1α (#ab51608, 1:200) were purchased from Abcam. The chromogenic procedures were conducted using DAB and hematoxylin. The stained slides were photographed by a bright-field microscope (Olympus). Positive reactions were defined as those showing brown signals, and the positive cells were analyzed by ImageJ software in five random fields. The microvessel density (MVD) was defined as CD31-positive cells per field of OC-2 KO tumor tissues compared with the control.

### Statistical Analysis

The experiments were performed independently at least three times and the data were represented as mean ± SD (standard deviation). Statistical analyses were conducted by one-way analysis of variance (ANOVA) with the least significant difference test using SPSS 19.0 software. *P* values < 0.05 (*) and < 0.01 (**) were considered statistically significant.

## Results

### Establishment of CRISPR/Cas9-Mediated OC-2 KO Ovarian Cancer Cell Lines

The double-strand DNA of the target area can be cleaved by Cas9 protein under the guidance of sgRNA. In the cleaved DNA, one or more bases (not a multiple of three bases) will be randomly inserted or deleted according to the insertion–deletion effect, leading to the frame shift mutation and gene knockout (30). The sgRNAs targeting OC-2 exon 1 were inserted into LentiCRISPRv2 at *Bsm*BI sites and the recombinant plasmid together with pMD2.G and pSPAX2 were transfected into SKOV3 and CAOV3 cells through lentivirus infection (Figure S1). Monoclonal OC-2 KO cell lines named O1D5, X-B10, J-E10, X-G1, and X-C1 (SKOV3 cells) and E1, G4, H8, G5, and G8 (CAOV3 cells) were randomly chosen from generated subclones. The lack of endogenous OC-2 protein was verified by Western blotting (Figure 1). Inhibition rates were listed as follows: O1D5 100%, J-E10 97%, X-B10 100%, X-G1 45%, and X-C1 50% (vs. SKOV3 control) and G4 99%, H8 98%, E1 60%, G5 35%, and G8 45% (vs. CAOV3 control). In Figure S2A, Sanger sequencing revealed homozygous and sgRNA-specific mutations to a reading frame shift. In SKOV3 cell lines, O1D5 was missing one base and X-B10 was added one base in exon 1 (sgRNA#1). In CAOV3 cell lines, G4 and H8 were deleted 56 and 221 bases (mixed sgRNAs). The deletion or insertion in these sequences was not a multiple of three bases, which could change the translation reading frame and knock out the OC-2 gene. The fragments cleaved by Cas9 protein were validated by Cruiser^TM^ to verify the cleavage efficiency of different sgRNAs (31). The results showed that the cleavage by mixed sgRNAs was more radical than single sgRNA, suggesting that the mixed lentivirus infection containing sgRNA#1–3 could enhance the knockout efficiency (Figure S2B). In summary, these findings strongly supported that the stable genetically modified OC-2 KO cell lines had been generated. OC-2 KO cell lines of O1D5, X-B10, J-E10, G4, and H8 with high inhibition rates were used at the following experiments.

The article "CRISPR/Cas9-Mediated OC-2 Editing Inhibits the Tumor Growth and Angiogenesis of Ovarian Cancer" was retracted in 2021. Reason: manipulated images.

**Figure 1:** Validation of OC-2 KO in SKOV3 and CAOV3 cells. The expression status of OC-2 was analyzed by Western blotting assay. From left to right, inhibition rates vs. SKOV3 control: O1D5 100%, J-E10 97%, X-B10 100%, X-G1 45%, and X-C1 50%; inhibition rates vs. CAOV3 control: G4 99%, H8 98%, E1 60%, G5 35%, and G8 45%. GAPDH served as loading control. The signal intensities were analyzed by ImageJ software.

### OC-2 KO Induced Apoptosis Activation and Inhibited the Proliferation, Migration, and Invasion of Ovarian Cancer Cells

To investigate the role of OC-2 in ovarian cancer progression, the stable OC-2 KO cell lines were subjected to serial experiments *in vitro*. At the loss of OC-2 expression, the apoptosis of SKOV3 and CAOV3 cells was up-regulated, with apoptosis rates of O1D5 35.3%, X-B10 21.4%, J-E10 29.9%, G4 15.5%, and H8 14%. Further, the expression of pro-apoptosis protein Bax was up-regulated while the anti-apoptosis protein Bcl-2 was down-regulated. The mitochondria-dependent caspase activation (Caspase-8) was observed in ovarian cancer cell lines in response to OC-2 knockout. Moreover, the expression levels of TP53 were decreased in both O1D5 and J-E10 cells (Figure 2). In the CCK-8 assay, the cell viability of OC-2 KO cell lines was significantly suppressed, with inhibition by 40–48% at 72 h (Figure 3A). In the wound-healing assay, the recovery of OC-2 KO cell lines was significantly decreased, with inhibition by 27.5–71.2% at 24 h (Figure 3B). In Transwell assays, the migration and invasion inhibition rates exceeded 41.7% in OC-2 KO cell lines (Figures 4A,B). Collectively, the results indicated that OC-2 played a key role in regulating the cell proliferation, migration, and invasion in ovarian cancer. When the expression of OC-2 was knocked out, the cell apoptosis of ovarian cancer was activated, leading to inhibition of tumor growth.

The article "CRISPR/Cas9-Mediated OC-2 Editing Inhibits the Tumor Growth and Angiogenesis of Ovarian Cancer" was retracted in 2021. Reason: manipulated images.

**Figure 2:** OC-2 KO induced apoptosis activation in SKOV3 and CAOV3 cells. The stained cells were detected by FACS, and the results were analyzed by FlowJo software. Up panel, representative images. Down panel, statistical analysis of apoptosis rate and qRT-PCR analysis of apoptosis markers. *P < 0.05, **P < 0.01.

**Figure 3:** OC-2 KO inhibited the cell viability of SKOV3 and CAOV3 cells. **(A)** Cells were cultured for the indicated time (0–72 h) and the cell viability was analyzed by CCK8 assay. **(B)** The monolayer cells were scraped in a straight line and the recovery of scratches was photographed at 24 h. The blank areas were measured by ImageJ software. Left panel, representative images. Right panel, statistical analysis of recovery data. Scale bars, 100 μm. *P < 0.05, **P < 0.01.

**Figure 4:** OC-2 KO significantly inhibited the migration and invasion of SKOV3 and CAOV3 cells. The cells suspended in 200 μl of basal DMEM were transferred into the upper chamber while 650 μl of DMEM with 10% FBS was added in the bottom. Matrigel was only used in the invasion assay. The migrated and invaded cells were fixed, stained, imaged, and calculated by ImageJ software in five random fields. **(A)** Cell migration was assayed by Transwell. **(B)** Cell invasion was analyzed by Transwell-Matrigel assay. Scale bars, 50 μm. Left panel, representative images. Right panel, statistical analysis of migrated and invaded data. **P < 0.01.

### OC-2 KO Down-Regulated the Expression of Pro-angiogenic Growth Factors and the Activation of Akt/ERK Pathways in Ovarian Cancer Cells

In the qRT-PCR assay, the mRNA levels of VEGFA, FGF2, and HIF-1α were decreased by 40–58%, 42–48%, and 49–56% in X-B10, O1D5, G4, and H8 cells, respectively. HGF was only down-regulated significantly in H8 cells (Figure 5A). Thus, OC-2 KO hampered the expression of pro-angiogenic growth factors at the transcriptional level. Next, assays of Western blotting and ELISA on the cell supernatant are needed to evaluate the secretion level. The Akt/ERK pathways are activated in numerous cellular events and closely related to cancer cell proliferation, metastasis, and angiogenesis (32, 33). According to the Western blotting analysis, the phosphorylation levels of ERK were decreased by 38–52% in X-B10 and O1D5 cells while the levels were decreased by 35–40% in G4 and H8 cells. The phosphorylation inhibition of Akt exceeded 55% in X-B10, O1D5, G4, and H8 cells (Figure 5B). The results indicated that OC-2 could positively regulate relevant pro-angiogenic growth factor expression and the Akt/ERK pathways to promote tumor growth and angiogenesis in ovarian cancer.

The article "CRISPR/Cas9-Mediated OC-2 Editing Inhibits the Tumor Growth and Angiogenesis of Ovarian Cancer" was retracted in 2021. Reason: manipulated images.

**Figure 5:** OC-2 KO down-regulated the expression of pro-angiogenic growth factors and the activation of Akt/ERK pathways in SKOV3 and CAOV3 cells. **(A)** qPCR analysis of expression levels of VEGFA, FGF2, HGF, and HIF-1α in X-B10, O1D5, G4, and H8 cells. **(B)** Western blotting analysis of the Akt/ERK pathways expression status in X-B10, O1D5, G4, and H8 cells. GAPDH served as loading control. The signal intensities were analyzed by ImageJ software. *P < 0.05, **P < 0.01.

### OC-2 Depletion Inhibited the Tumor Growth and Angiogenesis in the Xenograft Model

The BALB/c nude mice were inoculated with OC-2 KO cell lines to investigate the inhibitory effects on tumor growth and angiogenesis. As shown in Figures 6, 7, in SKOV3-bearing mice, OC-2 KO could significantly suppress tumor growth, with the inhibition exceeding 56% (O1D5 and X-B10) and the MVD was decreased by 71% (O1D5). In CAOV3-bearing mice, the tumor inhibition rates were 30–45% (G4 and H8) while the MVD was decreased by 62% (H8). In the sections of tumor tissues, the expression levels of OC-2, VEGFA, and HIF-1α were significantly down-regulated, with the inhibition exceeding 87%. Collectively, the results suggested that the tumor growth and angiogenesis were significantly inhibited when OC-2 was deleted, which might provide a potential target for ovarian cancer treatment.

**Figure 6:** OC-2 KO inhibited the tumor growth of SKOV3 and CAOV3 cells in the xenograft model. Mice (*n* = 3) were subcutaneously given injection of SKOV3, CAOV3, and OC-2 KO clones (1 × 10^6^ cells/mouse) in the right shoulder. From left to right, the stripped tumors, statistical analysis of tumor volume, and tumor weight. *P < 0.05, **P < 0.01.

**Figure 7:** OC-2 KO inhibited the tumor angiogenesis in the xenograft model of SKOV3 and CAOV3 cells. IHC staining was performed to analyze the expression levels of CD31, OC-2, VEGFA, and HIF-1α in tumor sections. The positive spots were indicated by red arrows and calculated by ImageJ software in five random fields. Up panel, representative images. Down panel, statistical analysis of positive expression data. Scale bars, 100 μm. *P < 0.05, **P < 0.01.

## Discussion

In this study, to investigate the function of OC-2 in ovarian cancer, the expression of OC-2 was completely deleted in SKOV3 and CAOV3 cells, and we successfully generated the OC-2 KO cell lines. In an *in vitro* experiment, we found that OC-2 KO could induce apoptosis activation, with up-regulation of pro-apoptosis protein Bax/Caspase-8 and down-regulation of anti-apoptosis protein Bcl-2. Moreover, the cell proliferation, migration, and invasion were significantly inhibited at the loss of OC-2. Further, the expression of pro-angiogenic growth factors VEGFA, FGF2, HGF, and HIF-1α and the activation of Akt/ERK pathways were down-regulated. In the xenograft model, OC-2 KO could inhibit the tumor growth and angiogenesis in BALB/c nude mice. The inhibition in O1D5 and X-B10 cells were more remarkable than G4 and H8 cells, which might be related to the expression levels of OC-2 in SKOV3 and CAOV3 cells. By using CRISPR/Cas9 technology, we figured out that the transcription factor OC-2 played a key role in the tumor growth and angiogenesis in ovarian cancer. As for J-E10 cells, although the missing 24 bases in exon 1 (mixed sgRNAs) were a multiple of 3 bases, the similar inhibition of tumor growth and angiogenesis was confirmed in this cell line. Since OC-2 was a transcription factor and the 24 bases of cleavage sites were in the same region relative to O1D5 and X-B10 cells, there might be a recognition region near the OC-2 cleavage sites that could bind and regulate downstream genes.

The article "CRISPR/Cas9-Mediated OC-2 Editing Inhibits the Tumor Growth and Angiogenesis of Ovarian Cancer" was retracted in 2021. Reason: manipulated images.

Tumor protein p53 (TP53) is defined as a tumor suppressor gene and is able to induce apoptosis activation. p53 mutants are the most common protein variants expressed in tumor cells, and many of them are oncogenic and anti-apoptotic (34). The expression of p53 was supposed to be up-regulated for promoting apoptosis but, in fact, down-regulated in O1D5 and J-E10 cells. However, the mitochondria-dependent Caspase-8 was activated due to the up-regulation of pro-apoptosis protein Bax and down-regulation of anti-apoptosis protein Bcl-2 (Figure 2). Although the Bcl-2 superfamily could be regulated in response to OC-2 KO, the molecular mechanism involved was still largely elusive.

The JASPAR database indicated that there were predicted binding sites of OC-2 on the promoter regions of VEGFA, FGF2, HGF, and HIF-1α (34). HIF-1α is able to induce tumor angiogenesis in a hypoxia environment through activating VEGFA transcription (35–37). Tacchin et al. found that HGF could not only increase the mRNA and protein levels of HIF-1α in HepG2 cells but also enhance the DNA binding activity of HIF-1α to modulate the VEGFA expression (38). Shi et al. reported that FGF2 induced HIF-1α expression by activating the Akt/ERK pathways in breast cancer (39). We hypothesized that FGF2 and HGF protein levels were decreased in OC-2 KO cell lines, which in turn inhibited the activation of HIF-1α to some extent. Then, the expression of VEGFA, the strongest pro-angiogenic growth factor, was down-regulated, destroying the angiogenesis networks (40). Importantly, the results of the qRT-PCR assay merely indicated that OC-2 positively regulated the expression of VEGFA, FGF2, HGF, and HIF-1α at the transcriptional level, but the accurate relationships among OC-2 and these pro-angiogenic growth factors required further investigation. Next, assays of Western blotting and ELISA on the cell supernatant should be conducted to evaluate the secretion level.

The article "CRISPR/Cas9-Mediated OC-2 Editing Inhibits the Tumor Growth and Angiogenesis of Ovarian Cancer" was retracted in 2021. Reason: manipulated images.

In numerous cellular events, the Akt/ERK pathways are activated by cytokines and growth factors via receptor-mediated phosphorylation cascade, including in tumor growth and angiogenesis (32, 33). OC-2 KO could inhibit the activation of Akt/ERK pathways, but the molecular mechanism that led to the reduced activity needed further investigation. To confirm the inhibitory effects, more analysis about phosphorylation cascade of Akt/ERK pathways in response to OC-2 KO and overexpression of OC-2 for recovery activation should be included in the following experiments. To confirm that the reduced phosphorylation of Akt or ERK was the cause of reduced viability, migration, and invasion, assays of phosphorylation inhibitors and recovery phosphorylation were more convincing. However, OC-2's mode of action remains to be fully understood in ovarian cancer cells. Whether there are other unknown pathways and mechanisms of OC-2 activity need to be further explored.

## Conclusions

By using CRISPR/Cas9 technology, we proved that OC-2 played a key role in cell apoptosis, proliferation, migration, invasion, and tumor angiogenesis of ovarian cancer. The tumor growth and angiogenesis were inhibited in response to OC-2 KO. Our results identified OC-2 as a unique target for developing broad-acting pro-apoptosis and anti-angiogenesis therapy in ovarian cancer. The CRISPR/Cas9-driven transcription factor knockout might help develop tumor gene therapy for reference in the future.

## Data Availability Statement

All datasets generated for this study are included in the article/Supplementary Material.

## Ethics Statement

The animal study was reviewed and approved by the Institutional Animal Care and Use Committee, Jinan University, Guangzhou, China.

## Author Contributions

ND, TL, LZ, and WZ designed and performed the experiments. LZ drafted and revised the manuscript. YZ and SZ participated in the experiments. BW was involved in resource collection. ND supervised this study. All authors read and approved the final manuscript.

The article "CRISPR/Cas9-Mediated OC-2 Editing Inhibits the Tumor Growth and Angiogenesis of Ovarian Cancer" was retracted in 2021. Reason: manipulated images.

## Conflict of Interest

The authors declare that the research was conducted in the absence of any commercial or financial relationships that could be construed as a potential conflict of interest.
